RETRACTED

# Long non-coding RNA TPT1-AS1 promotes cell growth and metastasis in cervical cancer via acting AS a sponge for miR-324-5p

**DOI:** 10.1186/s13046-018-0846-8

**Published:** 2018-07-25

**Authors:** Hui Jiang, Guanqun Huang, Nianzhang Zhao, Ting Zhang, Mengni Jiang, Yueming He, Xinke Zhou, Xianhan Jiang

**Affiliations:** 1 Department of Abdominal Oncology, The Fifth Affiliated Hospital of Guangzhou Medical University, Guangzhou, 510700 China; 2 Department of Gynaecology, The Fifth Affiliated Hospital of Guangzhou Medical University, Guangzhou, 510700 China; 3 Department of General Surgery, The Fifth Affiliated Hospital of Guangzhou Medical University, Guangzhou, 510700 China; 4 Department of Anesthesia, The Fifth Affiliated Hospital of Guangzhou Medical University, Guangzhou, 510700 China

**Keywords:** TPT1-AS1, Cervical cancer, miR-324-5p, SP1, EMT

## Abstract

**Background:**

Increasing studies confirmed that abnormal lncRNAs expression play a critical role in cervical cancer (CC) development and progression. LncRNA TPT1-AS1, a novel lncRNA, its role and underlying mechanisms involved in CC remain largely unknown.

**Methods:**

Colony formation, EdU and Transwell assays were used to determine colony formation, proliferation, migration and invasion in vitro. The subcutaneous tumor model and tail vein injection lung metastasis model were performed to check tumor growth and metastasis in vivo. Luciferase activity and RIP experiment were carried out to determine the interaction between miR-324-5p and TPT1-AS1.

**Results:**

We demonstrated for the first time that TPT1-AS1 expression was up-regulated in CC tissues and cell lines. High TPT1-AS1 was significantly correlated with adverse prognostic characteristics and poor survival. TPT1-AS1 overexpression and knockdown experiments revealed that TPT1-AS1 promoted cell colony formation, proliferation, migration, invasion and EMT progression of CC cells in vitro and in vivo. The underlying mechanism indicated that TPT1-AS1 functioned as an endogenous sponge for miR-324-5p in CC cells. Gain- and loss- experiment confirmed that miR-324-5p inhibited cell colony formation, proliferation, migration, invasion and EMT progression of CC cells, and mediated the biological effects of TPT1-AS1. Further investigations confirmed that SP1 was a direct target of miR-324-5p and mediated the effects of TPT1-AS1 and miR-324-5p in CC.

**Conclusions:**

We demonstrated for the first time that TPT1-AS1 as an oncogenic lncRNA in CC progression and as a potential target for CC cure.

**Electronic supplementary material:**

The online version of this article (10.1186/s13046-018-0846-8) contains supplementary material, which is available to authorized users.

RETRACTED

## Background

Cervical cancer (CC) is one of the most common malignant gynecologic cancers and the leading reason of cancer-associated mortality among female population [1, 2]. Despite great advancement in therapeutic approaches including surgery, radiotherapy and chemotherapy, a considerable patients’ long-term survival rate remains unsatisfactory due to recurrence and metastasis [3–5]. Hence, it’s urgent to explore the underlying biological mechanisms in the progress of CC and develop a better therapeutic intervention for CC.

Recently, non-coding RNAs, which contains microRNAs (miRNAs) and long non-coding RNAs (lncRNAs), have been recognized as novel candidates of signs or potential targets of treatment in multiple cancers [6–8]. Accumulating evidence reported that aberrant lncRNAs play critical roles in diverse biological courses including cellular differentiation, proliferation, apoptosis, migration, invasion and stem-cell biology [9–13]. For instance, Wang et al. showed that lncRNA CASC2 participated in tumor progression and exerted its inhibitory effects on hepatocellular carcinoma by CASC2/miR-367/FBXW7 pathway [7]. Upregulation of lncRNA SNHG12 increased cell growth and invasion in cervical cancer through acting as a sponge for miR-424-5p [14]. Recent studies demonstrated that lncRNA TPT1-AS1 was dysregulated in glioma [15]. However, the expression level and effects of TPT1-AS1 in CC remain largely unknown.

Emerging evidence indicates that microRNAs participate in many physiological and pathological processes [16–18]. miR-324-5p, a novel cancer-related miRNA, was dysregulated in many tumors [19–22]. miR-324-5p inhibits HCC invasion by counteracting ECM degradation through regulating ETS1 and SP1 [23]. Up-regulation of miR-324-5p suppressed cell growth and invasion of colorectal cancer cells by targeting ELAVL1 [24]. However, its role in CC remains unclear.

In the present research, we attempted to explore the expression, clinical importance, functions and potential mechanisms of TPT1-AS1 in CC. Gain- and loss-of-function analysis confirmed the biological function of TPT1-AS1 in vitro and in vivo on CC development. Finally, we demonstrated that TPT1-AS1 promoted cell proliferation, colony formation, migration and invasion via TPT1-AS1/miR-324-5p/SP1 axis in cervical cancer.

## Methods

### Clinical samples and cell culture

The matched CC tissues and corresponding non-cancer tissues were obtained in our hospital. Informed written consent was acquired from each patient and this program was approved by the Ethics Committee of our hospital in accordance with Helsinki Declaration. Human CC cells (C33A, SiHa, HeLa, CaSki, ME-180) and immortalized cervical epithelium NC104 (Chinese Academy of Sciences, Shanghai, China) were cultured in incubator (37 °C, 5% CO2), and cultured in RPMI1640 (Gibco, Grand Island, NY, USA) supplemented with 10% FBS (Gibco, Grand Island, NY, USA) and 1% penicillin-streptomycin (Invitrogen, CA, USA).

RETRACTED

### qRT-PCR

TRIzol reagent (Invitrogen, Carlsbad, CA) was used to isolate total RNA according to the manufacturer’s instructions. SYBR Premix Ex Taq II (TaKaRa, Dalian, China) was used to perform quantitative PCRs. qPCR primers were purchased from Genecopoeia (Guangzhou, China).

### Immunohistochemical (IHC) staining

We conducted the samples in a procedure by dewax, dehydrate and rehydrate. Primary antibody (1:100, Cell Signaling, Danvers, MA, USA) was used and incubating at 4 °C overnight. The biotinylated secondary antibodies (Goldenbridge, Zhongshan, China) was used to perform SP-IHC assays. The staining scores was evaluated by the positive intensity and average percentage for 6 independent fields.

### Western immunoblotting

RIPA lysis buffer (Pierce, Rockford, IL) was used to extract protein and BCA reagent (Rockford, IL, USA) was performed to quantify protein concentration. SDS-PAGE gel to separate the protein and detailed was performed as before [25].

### Transwell migration and invasion assay

The migration and invasion assays were performed using Transwell chamber (Millipore, Billerica, USA). The detailed was performed as previous studies [25].

### Colony assays and cell proliferation assays

Briefly, we plant cells at concentration 500 cells/well in six-well plate. After incubation for two weeks, we stained the colonies with 1% crystal violet and counted the number to quantify. EdU assays were conducted according to the protocols by manufacturer.

### In vivo experiments

We purchased 4–6-week BALB/c nude mice from the Centre of Laboratory Animals of The Fifth Affiliated Hospital of Guangzhou Medical University to conduct the subcutaneous model and the tail vein injection of lung metastatic model. We used hematoxylin and eosin (H&E) staining to check the lung metastatic foci after 3 weeks’ injection. We determined the subcutaneous tumor volume = length × width × width/2. We maintained the animals in standard conditions.

### Statistical analysis

All date is quantified as the Mean ± SD. The SPSS Version 13 (SPSS, Chicago, IL, USA) was conducted for the Pearson chi-square tests. A two-tailed Student’s t test was used to measure significance by GraphPad Prism 5 software (GraphPad Software, Inc., San Diego, CA, USA). *P* < 0.05 was considered to be statistically significant.

## Results

### Expression and clinical significance of TPT1-AS1 in CC

To confirm the expression level of TPT1-AS1 in CC, we firstly determined TPT1-AS1 expression in 40 randomly selected CC tissues and adjacent non-tumor tissues by qRT-PCR. Our results showed that TPT1-AS1 expression was significantly up-regulated in CC tissues compared to matched adjacent non-tumor tissues (*P* < 0.05, Fig. 1a). Furthermore, TPT1-AS1 expression in FIGO stage II was significantly higher than that in FIGO stage I (*P* < 0.05, Fig. 1b). Interestingly, TPT1-AS1 expression was up-regulated in CC with lymph node metastasis (LNM) compared with patients without LNM (NLNM) (*P* < 0.05, Fig. 1c). Moreover, the expression of TPT1-AS1 in a panel of CC cell lines were obviously increased compared to the immortalized cervical epithelial cell line (NC104) (*P* < 0.05, Fig. 1d). We determined the median cut-off = 0.62 to divide the patients into two subgroups. In clinical data, we determined that increased TPT1-AS1 expression was significantly associated with larger tumor size (*P* = 0.002), advanced FIGO stage (*P* = 0.005) and lymph node metastasis (*P* = 0.028) in CC (Table 1). In addition, Kaplan-Meier survival analysis revealed that the patients with high TPT1-AS1 expression had a poorer overall survival in CC (*P* < 0.05, Fig. 1e). These data indicated that TPT1-AS1 functions as an oncogene and correlates with the progression of CC.

RETRACTED

**Fig. 1:** lncRNA TPT1-AS1 was significantly up-regulated in CC and correlates with CC progression. **a** The expression level of TPT1-AS1 was detected in human CC tissues and matched adjacent normal tissues by qRT-PCR (*n* = 40). **b** Expression of TPT1-AS1 was increased in FIGO stage II relative to FIGO stage I (*n* = 20). **c** The expression of TPT1-AS1 in lymph node metastasis was significantly increased compared to that without lymph node metastasis (*n* = 8). **d** TPT1-AS1 expression in cervical cancer cell lines and an immortalized cervical epithelial cell line (NC104). **e** Kaplan-Meier curve of overall survival rate of cervical cancer patients with high TPT1-AS1 levels (*n* = 59) and low TPT1-AS1 levels (*n* = 56). *P < 0.05, **P < 0.01

**Table 1:** Clinical correlation of TPT1-AS1 expression in CC (*n* = 115)

Clinical parameters	Cases (n)	Expression level		*P* value (* *p* < 0.05)
		TPT1-AS1^high^(*n* = 59)	TPT1-AS1^low^(*n* = 56)	
Age(years)				
< 45 years	33	18	15	0.659
≥ 45 years	82	41	41	
FIGO stage				
I	67	27	40	0.005*
II	48	32	16	
Tumor size (cm)				0.002*
<4	63	24	39	
≥ 4	52	35	17	
LNM				0.028*
Negative	86	39	47	
Positive	29	20	9	
Vaginal invasion				0.752
Negative	91	46	45	
Positive	24	13	11	
Histology				0.866
Squamous	100	51	49	
Adenocarcinoma	15	8	7	
Parametrail extention				0.433
Negative	102	51	51	
Positive	13	8	5	

*FIGO* International Federation of Gynecology and Obstetrics, *LNM* lymph node metastasis

*Statistically significant by Pearson chi-square test

RETRACTED

### TPT1-AS1 promotes cell colony formation, proliferation, migration and invasion in vitro and in vivo

To observe the functional relevance of TPT1-AS1 in CC cells, we transfected C33A whose TPT1-AS1 was lowest with functional pcDNA/TPT1-AS1 and transfected CaSki who had highest TPT1-AS1 with specific shRNA (*P* < 0.01, respectively, Fig. 2a). Thereafter, Colony formation and Edu assays confirmed that TPT1-AS1 overexpression promoted cell colony formation and proliferation (*P* < 0.05, Fig. 2b, c). Transwell assays showed the migration and invasion were increased by TPT1-AS1 overexpression (*P* < 0.05, Fig. 2d, e). EMT has been recognized as key regulator of metastasis of CC. Therefore, we explored whether TPT1-AS1 regulated EMT process in CC cells. WB results showed that TPT1-AS1 overexpression significantly reduced the expression of epithelial marker E-cadherin and increased the mesenchymal marker Vimentin (*P* < 0.05, Fig. 2f). In contrary, TPT1-AS1 knockdown showed opposite effects in CaSki cells (*P* < 0.05, Fig. 2b-f). These findings indicated that TPT1-AS1 exerts as an important regulator in promotion of proliferation and EMT-mediated invasion of CC cells in vitro.

**Fig. 2:** TPT1-AS1 promotes cell colony formation, proliferation, migration, invasion and EMT progress in CC cells in vitro. **a** C33A and CaSki cells that were transfected with corresponding lncRNA vectors were subjected to qRT-PCR for TPT1-AS1 expression. Overexpression of TPT1-AS1 promoted cell colony formation (**b**), proliferation (**c**), migration (**d**) and invasion (**e**) in C33A cells, while down-regulation of TPT1-AS1 inhibited cell colony formation (**b**), proliferation (**c**), migration (**d**) and invasion (**e**) in CaSki cells. **f** Western blot analysis of EMT-related markers expression in the presence and absence of TPT1-AS1. *n* = six independent experiments. *P < 0.05, **P < 0.01

To explore the potential functions of TPT1-AS1 in vivo, we firstly used the subcutaneous tumor model to conduct that TPT1-AS1 overexpression significantly promoted tumor growth, while TPT1-AS1 knockdown inhibited the tumor growth of CC cells in mice (*P* < 0.05, Fig. 3a, Additional file 1: Figure S1). Moreover, we established a lung metastasis model by tail vein injection to measure metastatic potential in vivo. Our data showed that TPT1-AS1 overexpression in C33A cells increased the lung metastasis while TPT1-AS1 knockdown reduced the lung metastasis of CaSki cells (*P* < 0.05, Fig. 3b). In addition, we used Ki67 staining which is a marker of proliferation to measure the proliferative activity in the xenografted tissues. As expect, TPT1-AS1 overexpression increased the Ki67 positive staining cells and reduced the number of positive cells after TPT1-AS1 knockdown (*P* < 0.05, Fig. 3c). Moreover, in lung metastasis sections and subcutaneous tumor tissues, TPT1-AS1 overexpression increased Vimentin expression and reduced E-cadherin expression (Fig. 3d, Additional file 2: Figure S2), while TPT1-AS1 knockdown showed opposite phenomenon (Fig. 3d, Additional file 2: Figure S2). Furthermore, in clinical CC tissues, we found that E-cadherin expression in TPT1-AS1 high expressing CC tissues was lower than that in low expressing cases. Conversely, the expression of Vimentin in the TPT1-AS1 high expression group was markedly higher than that in low expression group (*P* < 0.05, respectively, Fig. 3e). Taken together, we demonstrated that TPT1-AS1 promoted tumor growth and metastasis of CC in vitro and in vivo.

RETRACTED

**Fig. 3:** TPT1-AS1 promotes tumor growth and metastasis in vivo*.* **a** Tumor growth curve revealed that TPT1-AS1 overexpression significantly promoted, while TPT1-AS1 knockdown inhibited tumor growth in vivo (*n* = 5). **b** Representative HE staining of lung metastases in TPT1-AS1 overexpression or knockdown cells (*n* = 5). **c** Tumor nodules were subjected to immunohistochemical staining for Ki-67 assays and quantitative analysis. Representative immunostaining assays revealed that TPT1-AS1 overexpression significantly increased the number of Ki-67 positive cells. However, the percentage of Ki-67 positive cells in tumors arising from the TPT1-AS1 knockdown group was significantly lower than that in the negative control group. **d** Immunohistochemistry of E-cadherin and Vimentin were showed and compared between tissues of respective TPT1-AS1 expression level. **e** Immunohistochemistry of E-cadherin and Vimentin were showed and compared between TPT1-AS1 high expressing CC tissues (*n* = 59) and TPT1-AS1 low expressing cases (*n* = 56). *P < 0.05

### TPT1-AS1 functions AS competing endogenous RNA and sponges miR-324-5p in CC cells

Previous studies reported that lncRNA could act as a competing endogenous RNA (ceRNA) or a molecular sponge to interact with miRNAs and participate the physiological and pathological process. The program StarBase v2.0 (http://starbase.sysu.edu.cn/) was used to predict potential lncRNA-miRNA interactions, and we found that TPT1-AS1 has a putative binding site for the seed sequence of miR-324-5p (Fig. 4a). Here, we report that TPT1-AS1 was localized preferentially in the cytoplasm as determined by FISH experiment (Additional file 3: Figure S3). TPT1-AS1 overexpression decreased miR-324-5p expression in C33A cells while TPT1-AS1 knockdown increased miR-324-5p in CaSki cells (*P* < 0.05, Fig. 4b). Moreover, our data showed that miR-324-5p was inversely correlated with TPT1-AS1 expression in CC tissues (*r* = − 0.8877, *P* < 0.001, Fig. 4c). Dual-luciferase reporter assays revealed that miR-324-5p inhibited luciferase activity in the TPT1-AS1 wild-type reporter gene but not in the mutant type (Fig. 4d). Moreover, RIP experiments showed that TPT1-AS1 and miR-324-5p were preferentially enriched in Ago2-containing microribonucleoproteins (miRNPs) relative to control IgG (Fig. 4e). Subsequently, we performed pull-down assay using biotin-labeled specific TPT1-AS1 probe. Our results showed that miR-324-5p obtained a great enrichment in the TPT1-AS1 pull down pellets compared with negative control group (*P* < 0.05, Fig. 4f). Taken together, these findings indicated that miR-324-5p was a downstream target of TPT1-AS1 in CC cells.

RETRACTED

**Fig. 4:** miR-324-5p was a target of TPT1-AS1 in CC. **a** Bioinformatics analysis showed that miR-324-5p could directly target 3′-UTR of TPT1-AS1-wild type (WT). TPT1-AS1-mutant (Mut) means mutation of binding sites in the 3′-UTR of TPT1-AS1. **b** Real-time PCR showed that TPT1-AS1 could negatively regulate miR-324-5p expression in CC cells. **c** Pearson correlation analysis revealed that an obvious negative association between miR-324-5p and TPT1-AS1 expression in CC tissues. **d** Dual luciferase reporter assays showed that miR-324-5p could negatively regulate the luciferase activity of TPT1-AS1-WT, rather than TPT1-AS1-Mut. **e** The association between TPT1-AS1, miR-324-5p and Ago2 was ascertained by analyzing C33A cell lysates using RNA immunoprecipitation with an Ago2 antibody. Real-time PCR was used to detect the TPT1-AS1 level change in the substrate of RIP assay in miR-324-5p-overexpressing CC cells. **f** Detection of TPT1-AS1 using real-time PCR in the sample pulled down by biotinylated TPT1-AS1 and negative control (NC) probe. Detection of miR-324-5p using real-time PCR in the same sample pulled down by biotinylated TPT1-AS1 and NC probe. *P < 0.05, **P < 0.01

### miR-324-5p served as tumor suppressor in CC

To explore the expression level of miR-324-5p in CC, we performed qRT-PCR to determine miR-324-5p in CC tissues and cells. Our data showed that miR-324-5p was down-regulated in CC tissues compared to adjacent non-tumor tissues (*P* < 0.05, Fig. 5a). Moreover, miR-324-5p was reduced in a panel of CC cell lines compared with NC104 cells (*P* < 0.05, Fig. 5b). To confirm the biological function of miR-324-5p on CC, we detected cell colony formation, proliferation, migration, and invasion capacities of CC cells after miR-324-5p overexpression or inhibition (*P* < 0.05, Fig. 5c). As shown in Fig. 5d-h, the cell colony formation, proliferation, migration, invasion and EMT progress was inhibited by miR-324-5p overexpression, while miR-324-5p knockdown showed opposite effects on CC cells (*P* < 0.05, Fig. 5d-h). These data indicated that miR-324-5p serves as a tumor suppressor in CC.

RETRACTED

**Fig. 5:** miR-324-5p served as tumor suppressor in CC. **a** qRT-PCR analysis of TPT1-AS1 expression in CC tissues and normal adjacent non-tumor tissue samples. **b** Expression levels of TPT1-AS1 were evaluated by qRT-PCR in normal cervical epithelium cell and CC cell lines. **c** CaSki and C33A cells that were transfected with corresponding miRNA vectors were subjected to qRT-PCR for miR-324-5p expression. Overexpression of miR-324-5p inhibited cell colony formation **d**, proliferation (**e**), migration (**f**), invasion (**g**) and EMT process (**h**) in CaSki cells, while down-regulation of miR-324-5p promoted cell colony formation (**d**), proliferation (**e**), migration (**f**), invasion (**g**) and EMT process (**h**) in C33A cells. *P < 0.05, **P < 0.01

### miR-324-5p reversed the promoting effects of TPT1-AS1 on CC cells

To dissect the importance of miR-324-5p binding in TPT1-AS1-promoting CC progression, we ectopically expressed miR-324-5p in stable TPT1-AS1 overexpressing C33A cells or transfected miR-324-5p antagomir to TPT1-AS1 knockdown CaSki cells (*P* < 0.05, Fig. 6a). We found that overexpression of miR-324-5p attenuated the promoting effect on cell colony formation, proliferation, migration and invasion and EMT process of CC (*P* < 0.05, Fig. 6b-f). Moreover, transfection with antagomir miR-324-5p rescued the inhibitory effect of TPT1-AS1 knockdown on cell colony formation, proliferation, migration and invasion and EMT process (Fig. 6b-f). Moreover, our data showed that miR-324-5p knockdown increased the SP1 expression, which abolished the effects of sh-TPT1-AS1-induced SP1 down-regulation in CaSki cells (*P* < 0.05, Additional file 4: Figure S4). These findings indicated that TPT1-AS1 promotes CC cell colony formation, proliferation, migration, invasion and EMT process in part via competitively binding with miR-324-5p.

**Fig. 6:** Restoration of miR-324-5p expression reversed the effects of TPT1-AS1 on CC cells. **a** TPT1-AS1-overexpressing C33A cells that were transfected with empty vector (miR-control) or miR-324-5p overexpression vector were subjected to qRT-PCR for miR-324-5p. TPT1-AS1-suppressive CaSki cells that were transfected with anti-miR-324-5p were subjected to qRT-PCR for miR-324-5p. miR-324-5p restoration abrogated the effects of TPT1-AS1 overexpression on cell colony formation (**b**), proliferation (**c**), migration (**d**), invasion (**e**) and EMT process (**f**) of C33A cells. miR-324-5p knockdown reversed the suppressive effects of TPT1-AS1-AS1 knockdown in CaSki cells (**b**-**f**)

RETRACTED

### miR-324-5p directly targeted SP1 in CC cells

To investigate the underlying mechanism by which miR-324-5p exerted its effects on CC cells, we searched public database to select candidate target of miR-324-5p and found SP1 3’-UTR contains binding sequence (Fig. 7a). Previous studies confirmed that SP1 is an oncogene and promotes migration, invasion in CC cells [26, 27]. To validate that miR-324-5p could interact with SP1 3’-UTR, we performed luciferase reporter assays and found miR-324-5p overexpression significantly reduced luciferase activity of wt SP1 3’-UTR, while miR-324-5p knockdown increased luciferase activity of SP1 3’-UTR (*P* < 0.05, Fig. 7b). However, miR-324-5p didn’t change the luciferase activity of mt SP1 3’-UTR (Fig. 7b). Moreover, qRT-PCR and WB also showed that miR-324-5p overexpression significantly inhibited, while miR-324-5p knockdown increased the mRNA and protein of SP1 in CC cells (*P* < 0.05, respectively, Fig. 7c, d). These data showed that SP1 was a downstream target of miR-324-5p. Moreover, we explored the correlation between miR-324-5p and SP1 in CC. Our data showed that both SP1 mRNA and protein expression in high miR-324-5p group were significantly lower than that in low miR-324-5p in CC (*P* < 0.05, Fig. 7e, f). Our IHC results showed similar results in CC tissues (Fig. 7g). Notably, miR-324-5p expression was inversely correlated with the SP1 mRNA in CC tissues (*r* = − 0.8412, *P* < 0.001, Fig. 7h). These findings conclude that SP1 was a downstream of miR-324-5p in CC.

**Fig. 7:** SP1 is a direct target of miR-324-5p in CC cells. **a** miR-324-5p and its putative binding sequences in the 3’-UTR of SP1. The mutant binding site was generated in the complementary site for the seed region of miR-324-5p. **b** miR-324-5p overexpression significantly suppressed, while miR-324-5p loss increased the luciferase activity that carried wild-type (wt) but not mutant (mt) 3’-UTR of SP1. miR-324-5p overexpression reduced the expression of SP1 mRNA (**c**) and protein (**d**) in CaSki cells and miR-324-5p knockdown increased the level of SP1 mRNA (**c**) and protein (**d**) in C33A cells. **e-g** The expression of SP1 in miR-324-5p high-expressing tumors was significantly lower than that in miR-324-5p low-expressing tumors, as determined by qRT-PCR (**e**), immunoblotting (**f**) and IHC (**g**). **h** An inverse correlation between the levels of miR-324-5p and SP1 mRNA was observed in CC tissues. *P < 0.05

RETRACTED

### Restoration of SP1 expression partially reversed the promotive effects of TPT1-AS1 and tumor-suppressive roles of miR-324-5p in CC cells

We firstly validate that TPT1-AS1 regulated SP1 expression. qRT-PCR and WB showed that TPT1-AS1 positively regulated SP1 mRNA and protein expression in CC cells (*P* < 0.05, respectively, Fig. 8a, b). To further confirm that the effects of TPT1-AS1 and miR-324-5p on CC is dependent on regulation of SP1 expression, we restored SP1 expression in CaSki-sh-TPT1-AS1 or CaSki-miR-324-5p cells by SP1 plasmids, or knockdown SP1 expression in C33A-TPT1-AS1 or C33A-anti-miR-324-5p by a specific siRNA (*P* < 0.05, Fig. 8c). Restored SP1 expression eliminated the inhibitory effects on colony formation, proliferation, migration, invasion and EMT progress induced by TPT1-AS1 knockdown or miR-324-5p overexpression (*P* < 0.05, respectively, Fig. 8d-h). By contrast, SP1 knockdown abolished the promotive functions on CC cells by TPT1-AS1 overexpression or miR-324-5p knockdown (*P* < 0.05, respectively, Fig. 8d-h). Therefore, we demonstrated that SP1 was a downstream mediator of TPT1-AS1/miR-324-5p axis in CC.

**Fig. 8:** Modulation of SP1 partially abolishes TPT1-AS1 or miR-324-5p-mediated cellular processes in CC. TPT1-AS1 overexpression increased the expression of SP1 mRNA (**a**) and protein (**b**) in C33A cells and TPT1-AS1 knockdown reduced the level of SP1 mRNA (**a**) and protein (**b**) in CaSki cells. **c** miR-324-5p-overexpressing or TPT1-AS1-suppressive CaSki cells that were transfected with empty vector (EV) or SP1 overexpression plasmid were subjected to western blot for SP1. miR-324-5p-suppressive or TPT1-AS1-overexpressing C33A cells that were transfected with scrambled siRNA or SP1 siRNA were subjected to western blot for SP1. SP1 restoration abrogated the effects of miR-324-5p overexpression or TPT1-AS1 knockdown on cell colony formation (**d**), proliferation (**e**), migration (**f**), invasion (**g**) and EMT process (**h**) of CaSki cells. SP1 knockdown reversed the promotive effects of miR-324-5p knockdown or TPT1-AS1 overexpression in C33A cells (**d**-**h**). *P < 0.05

## Discussion

Numerous lncRNAs are aberrantly expressed in CC and play critical roles in the onset and progression of CC by acting as either tumor suppressor or oncogene [28, 29]. Therefore, it may provide valuable therapeutic targets in the strategy for patients’ treatment to investigate the biological function and underlying mechanisms of lncRNAs in CC. In current research, we demonstrated for the first time that lncRNA TPT1-AS1 expression was up-regulated in CC tissues and cell lines. Its high expression was significantly associated with adverse clinical features, including FIGO stage, tumor size and lymph node metastasis and worse prognosis. These findings indicated that TPT1-AS1 serve as an oncogene and play critical role in CC progression.

RETRACTED

To elucidate the biological function of TPT1-AS1 in CC, we performed gain- and loss-of-function experiment and showed that TPT1-AS1 overexpression promoted cell colony formation, proliferation, migration, invasion and EMT progress in vitro and in vivo. Moreover, we furthermore confirmed TPT1-AS1 was remarkably correlated with EMT markers in CC tissues. These data suggested that TPT1-AS1 play an important role in the biological function of CC development. Recently, accumulating studies reported that lncRNAs act as a ceRNA or miRNA sponge via interacting with miRNAs and suppressing their effects [30]. Therefore, we assumed that TPT1-AS1 serve as a miRNA sponge in CC. To confirm the hypothesis, we conducted bioinformatic analysis and miR-324-5p contains the binding site of TPT1-AS1. Gain- and loss- experiment showed that TPT1-AS1 negatively regulated the expression of miR-324-5p in CC cells. In CC tissues, TPT1-AS1 existed an inverse correlation with miR-324-5p. Moreover, to confirm TPT1-AS1 could directly bind with miR-324-5p, luciferase reporter gene and anti-Ago2 RIP revealed that TPT1-AS1 directly targeted miR-324-5p in CC cells. In addition, we also confirmed that miR-324-5p was down-regulated in CC tissues and cell lines. Functional experiment showed that miR-324-5p inhibited cell colony formation, proliferation, migration, invasion and EMT progress in CC cells. Recent studies demonstrated that miR-324-5p play a key role in tumor progression [31]. What’s more, rescue experiments in vitro experiments manifested that miR-324-5p was a mediator for TPT1-AS1 in CC cells. These data strongly demonstrated that TPT1-AS1 may act as a sponge for miR-324-5p in CC cells.

Furthermore, we attempted to explore the downstream target of miR-324-5p in CC cells, which may mediate TPT1-AS1/miR-324-5p axis. Then, bioinformatics tools combined with previous studies were employed for comprehensive analysis. According to the bioinformatics database, we found that SP1, a critical oncogene that regulated multiple cellular process in CC [32], may be one of the candidate target o miR-324-5p. Previous studies confirmed that SP1 is a target of miR-324-5p in HCC cells [23]. Luciferase reporter assays indicated that miR-324-5p directly targeted SP1 3’UTR. In addition, qRT-PCR and Western blot showed that miR-324-5p negatively regulated the expression of SP1 mRNA and protein. In CC tissues, the mRNA and protein of SP1 in high miR-324-5p tissues was lower than that in low miR-324-5p tissues. Moreover, miR-324-5p showed a negative relationship with SP1 in CC tissues. Finally, to investigate the role of SP1 in TPT1-AS1/miR-324-5p axis, we performed rescue experiment that reversed SP1 expression both abolished the biological function of TPT1-AS1 and miR-324-5p in CC cells. Previous studies demonstrated that SP1 could bind to the Snail promoter, which is a transcript factor of EMT-related protein, contribute to the tumor metastasis [33, 34]. SP1 also affects the proliferation of cervical cancer in different mechanisms [26, 35]. These findings suggest that SP1 mediated the TPT1-AS1/miR-324-5p-induced biological function on CC cells.

RETRACTED

In conclusion, our study demonstrated for the first time that TPT1-AS1 is up-regulated in CC tissues and cells. Its high expression is associated with malignant clinical features and poor prognosis in CC patients. Gain- and loss-of-function confirmed that TPT1-AS1 promoted cell colony formation, proliferation, migration, invasion and EMT progress via miR-324-5p/SP1 axis, which could be a valuable and promising therapeutic target for CC treatment.

## Conclusions

To conclude, our data offer the promising evidence that TPT1-AS1 overexpression acts as a predictor for indicating adverse clinical features and poor prognosis of CC patients. TPT1-AS1 facilitates CC cell colony formation, proliferation, migration, invasion and EMT progress in vitro and in vivo. MiR-324-5p was identified as not only a target but also a functional mediator of TPT1-AS1 in CC cells. miR-324-5p suppressed colony formation, proliferation, migration, invasion and EMT process of CC cells by directly targeting SP1. Restoration SP1 reversed the biological function of TPT1-AS1 and miR-324-5p on CC cells. To conclude, TPT1-AS1/miR-324-5p/SP1 axis suppressed cellular process of CC cells. These findings will improve understanding of mechanism involved in cancer progression and provide novel targets for the molecular treatment of CC.

## Additional files

Additional file 1: Figure S1. TPT1-AS1 promotes tumor growth in vivo*.* (A) Tumor weight revealed that TPT1-AS1 overexpression significantly promoted, while TPT1-AS1 knockdown inhibited tumor growth in vivo. (TIF 976 kb)

Additional file 2: Figure S2. Immunohistochemistry of E-cadherin and Vimentin were showed and compared between tissues of respective TPT1-AS1 expression level in subcutaneous tumor tissues. (TIF 1878 kb)

Additional file 3: Figure S3. FISH was used to confirm TPT1-AS1 location in CaSki cells, using probes for TPT1-AS1, DAPI for nuclear staining. (TIF 310 kb)

Additional file 4: Figure S4. miR-324-5p knockdown increased the SP1 expression, which abolished the effects of sh-TPT1-AS1-induced SP1 down-regulation. (TIF 100 kb)

RETRACTED

## Abbreviations

3’-UTR: 3′-untranslated region
CC: Cervical cancer
EMT: Epithelial-mesenchymal transition
H&E: Hematoxylin and eosin
IHC: Immunohistochemistry
lncRNA: Long non-coding RNA
miRNAs: microRNAs
qRT-PCR: Real-time quantitative reverse transcription polymerase chain reaction
RIP: RNA immunoprecipitation
SP1: Specificity protein 1
